# Meta-Analysis of the Association Study between Allergic Rhinitis and HLA-II Gene (DQB1) in Northern China

**DOI:** 10.1155/2021/4356770

**Published:** 2021-09-23

**Authors:** Jie Wang

**Affiliations:** College of Nursing, Bengbu Medical College, Bengbu 233030, Anhui, China

## Abstract

**Objective:**

To explore the association between allergic rhinitis and HLA-II gene (DQB1) in the Chinese population.

**Methods:**

The literature studies related to allergic rhinitis and HLA-II gene (DQB1) in the Chinese population were searched, and those that did not meet the requirements were excluded. The consistency was checked by using RevMan 4.1 software.

**Results:**

The HLA-II gene (DQB1) may be a risk gene for patients with allergic rhinitis in Northern China (*P* < 0.01).

**Conclusion:**

Allergic rhinitis in China was associated with the HLA-II gene (DQB1).

## 1. Introduction

Allergic rhinitis (AR) is a complex disease with a high incidence. The factors leading to the disease are very complex. It is now believed that the incidence of AR has been increasing over the past few decades due to the interaction of genetic variation and genetic environment, affecting the lives of more than 1.4 billion people [1, 2]. AR is characterized by a severe response to allergens, resulting in increased airway secretion, increased sensitivity, nasal congestion, itching, runny nose, and sneezing symptoms. AR seriously affects the quality of life of patients. It places a significant burden on the health maintenance costs of individuals and on the medical resources of the society. At present, the pathogenesis of AR has not been fully clarified. However, many scholars believe that unbalanced T helper cell 1 (Th1)/Th2 immune response and elevated levels of immunoglobulin E (IgE) to inhaled allergens are important pathogenesis [3].

AR is an immunoglobulin E*-* (IgE-) mediated immune-related nasal mucosal inflammatory response. Studies now show that there are many pathogenic factors such as environment and genes. It is a multigene complex disease. In the HLA gene family, because the function of the HLA-II gene is closely related to the initial manifestations of allergic rhinitis, related research has received widespread attention [1]. Shiina et al. [4] studied the genetic model of the HLA-II gene (HLA-DRB1 and HLA-DQB1) and related diseases. The meta-analysis of the disease shows that the HLA-DQB1 gene is related to specific IgE-mediated allergic diseases. Other scholars [5–9] have also confirmed the correlation between HLA-DQB1 gene polymorphisms and allergic diseases. However, there are many members of the HLA allele family, which are quite complex. The significant linkage disequilibrium and dominant inheritance characteristics of genes make it difficult to explore. This article explores the correlation between HLA genes and diseases [10].

## 2. Materials and Methods

Meta-analysis: correlation between allergic rhinitis and HLA-DQB1 gene in the Chinese population in the Chinese Biomedical Literature Database and China HowNet Medical Search (CBM 2005–2019) (Time: January 2002 to January 2019). Search terms use “allergic rhinitis” and “HLA” or “allergic rhinitis and human leukocyte antigen”; search Medline uses “allergic rhinitis” and “human leukocyte antigen” or “gene”; search EM-Base uses “allergic Rhinitis or allergic rhinitis” and “hitocompatibility.” Inclusion criteria were as follows: (1) all cases involving the HLA-II gene (DQB1) in the population in Northern China. (2) All studies included case groups and control groups. The case group was patients with allergic rhinitis, for any reason, and all met the revised classification criteria for allergic rhinitis. The control group was a healthy population and had no blood relationship with the patients. (3) The age and sex of the control group and the case group were basically the same. (4) If there were multiple articles in the same sample population, the latest published article was selected as the research object. Exclusion criteria were as follows: (1) duplicate reports and unclear data descriptions; (2) overseas Chinese.

Statistical analysis was performed using the meta-analysis software package RevMan 4.1. Heterogeneity was calculated by using the *Q*-test statistics. The OR values of the studies included in the meta-analysis were plotted on the abscissa, and the standard error was used as the ordinate to plot the inverted funnel. Its symmetry was observed, and the impact of publication bias was evaluated.

## 3. Results

Through machine inspection, a total of 26 articles were retrieved. Based on the title, abstract, and original text, articles that clearly did not meet the inclusion criteria were excluded. Of these samples, 26 were excluded, including duplicate reports. The basic information of the meta-analysis literature and the quality evaluation of each literature study were included in the case-control study. The object was Chinese, and the diagnosis was clear. The original data provided the OR value and its 95% confidence interval (CI). They contained sufficient information for comparing the case groups. We compared the distribution of HLA-DQ alleles with the control group. There was no statistically significant difference in age and gender distributions between the case group and the control group. Other basic information and the concrete DQB1 susceptibility gene locus with the statistical *P* value by contrast with the control group are shown in Table 1.

Evaluation of publication bias: by observing the inverted funnel plot of each HLA-DQ allele in the meta-analysis, it was found that the symmetricalness of the inverted funnel plot is DQB1 ^*∗*^ 06 : 01 : 01 and DQB1 ^*∗*^ 0602; their meta-analysis results' published bias were smaller. The inverted funnel plots of DQB1 ^*∗*^ 04 have poor symmetry, and their meta-analysis results have a large publication bias.

## 4. Discussion

HLA is located in the 6p21.3 region of the short arm of human chromosome 6, with a total length of about 3600–4000 kb. It is divided into HLA-I, II, and III genes, most of which are related to the immune response. Among them, HLA-I and HLA-II genes are mainly involved in antigen presentation. The human major histocompatibility complex (MHC) contains 128 functional genes, of which 39.8% are related to the immune system. Therefore, 39.8% of genes may be directly or indirectly related to the occurrence of many autoimmune diseases [14]. The HLA-II gene includes at least three subregions of HLA-DR, DQ, and DP. HLA-DQ polymorphisms are known to be most closely related to the production of SLE autoantibodies.

Meta-analysis has a scientific and reasonable side, but it also has certain limitations and problems. Because meta-analysis is a descriptive analysis, there are confusion biases, errors reported in the literature, and some shortcomings of the analysis method, but meta-analysis should be relatively correct and applied to medical practice and scientific research [15]. Meta-analysis must follow a specified methodology and procedure, emphasize extensive searches and clear literature inclusion and exclusion criteria, and use quantitative methods based on rigorous quality assessments of included studies to quantitatively combine them to minimize deviation. The biggest disadvantage of meta-analysis is that the research objects are not correctly combined. In gene association analysis, because the diagnosis of the disease is simple and standard, most methods use the more advanced PCR-SSP, PCR-SSO, and PCR-RFLP methods. Genotypes are easier to identify. This study is largely unaffected by this factor.

Two alleles of HLA class II genes, DRB1 and DQB1, are significantly associated with allergen-specific IgE responses [4]. A close association between HLA class II alleles (DR, DQ, and DP) and specific IgE responses to airborne pollen and HDM allergens was reported [5–8]. Rich genetic polymorphisms of HLA-DRB1 and HLA-DQB1 can be observed in allergic diseases [16, 17].

The results of this meta-analysis suggest that DQB1 ^*∗*^ 06 : 01 : 01 and DQB1 ^*∗*^ 0602 may be risk genes for SLE patients in the Chinese population.

This investigation and research included different factors of Artemisia pollen allergic rhinitis; Xinjiang Uygur and Han allergic rhinitis; dust mite allergic rhinitis; and allergice rhinitis of different nationalities that causes allergic rhinitis in the Chinese population.

## Figures and Tables

**Table 1:** The basic information and the concrete DQB1 susceptibility gene locus with the statistical *P* value by contrast with the control group.

Numbering	Study	Population	Sample content	Control group	Susceptibility	*P*
1	Zhao et al. [11]	North of China	71	92	DQB1 ^*∗*^ 06 : 01 : 01	≤0.001
2	Zhao et al.	North of China	71	92	DQB1 ^*∗*^ 05 : 02 : 01	0.024
3	Zhao et al.	North of China	71	92	DQB1 ^*∗*^ 05 : 03 : 01	0.020
4	Zhao et al.	North of China	71	92	DQB1 ^*∗*^ 06 : 02 : 01	0.011
5	Zhao et al.	North of China	71	92	DQB1 ^*∗*^ 06 : 04 : 01	0.044
6	Cui et al. [12]	Uighur	50	50 (Han)	DQB1 ^*∗*^ 03	0.105
7	Cui et al.	Uighur	50	50 (Han)	DQB1 ^*∗*^ 02	0.575
8	Cui et al.	Uighur	50	50 (Han)	DQB1 ^*∗*^ 06	0.276
9	Cui et al.	Uighur	50	50 (Han)	DQB1 ^*∗*^ 05	0.010
10	Cui et al.	Uighur	50	50 (Han)	DQB1 ^*∗*^ 04	1.000
11	Xing et al. [13]	Beijing area	41	41	DQB1 ^*∗*^ 0602	<0.01

## Data Availability

The data used to support the findings of this study are available upon request to the author.
